# Phosphate and Nitrate Removal from Coffee Processing Wastewater Using a Photoelectrochemical Oxidation Process

**DOI:** 10.1155/2022/4382491

**Published:** 2022-09-19

**Authors:** Firomsa Bidira, Zerihun Asmelash, Seifu Kebede, Abreham Bekele

**Affiliations:** ^1^Faculty of Civil and Environmental Engineering, Jimma Institute of Technology, Jimma University, P.O. Box 378, Ethiopia; ^2^School of Chemical Engineering, Jimma Institute of Technology, Jimma University, P.O. Box 378, Ethiopia

## Abstract

Water quality, whether utilized for home, irrigation, or recreational reasons, is crucial for health in both developing and developed countries around the world. For the treatment of nitrate (NO_3_) and phosphate (PO_3_) from coffee processing wastewater, photoelectrochemical oxidation was used. This process is mainly used to destroy pollutants through the production and use of powerful oxidized species such as hydroxyl radical (OH). It investigated the effects of Uv/H_2_O_2_ on electrochemical processes and the effects of various parameters such as pH, time, current, and electrolytes. The results were calculated and analyzed using response surface methodology and Microsoft Excel. Hybrid photoelectrochemical oxidation (PECO) using UV and hydrogen peroxide (UV/H_2_O_2_) methods removed nitrates (99.823%) and phosphates (99.982%). These results were obtained with pH 7, current 0.40 amperes, and 1.5 g calcium chloride after 40 minutes of electrolysis. CaCl_2_ was more effective in removing organic compounds from coffee processing wastewater. An analysis of variance (ANOVA) with a 95% confidence limit was used to determine the significance of the independent variable.

## 1. Introduction

The industrialization and development of manufacturing processes have increased the amount of sewage in the environment that causing water pollution [1]. Wastewater treatment is becoming an increasingly important aspect of industrial production. Coffee is the most popular drink in the world, with millions of people drinking it every day [2]. Ethiopia is one of the largest producers of million tons of coffee per year. The coffee processing technique can be either dry or wet types. Coffee processing companies produce a high pollutant load with wastewater since they use the largest water and produce a large volume of wastewater. The wastewater from the coffee processing unit has high concentrations of organic matter, nutrients, suspended particles, and extremely, BOD_5_, COD, N, P, TDS, and TSS. These components are all important in coffee wastewater because they are related to the pH, temperature, turbidity, and electrical conductivity of wastewater [3]. Wet treatment systems use large amounts of water and therefore produce large amounts of contaminated sewage. It has traditionally been easily discharged into nearby streams and rivers [4]. This is because the quality of coffee beans deteriorates hours after they are harvested on the farm. This is because coffee beans require immediate and rapid processing [5]. To remove the cherries from the coffee, a lot of water is needed throughout the processing [6]. The effluent mainly comes from coffee bean washing and floor washing. On the one hand, sugar-rich digested water ferments rapidly with the help of enzymes from coffee cherry bacteria. On the other hand, depending on the treatment method, there is water from fermentation and washing and viscous wastewater from mechanical expectorants [7]. According to [8], coffee processing wastewater composition coffee Arabica contains 32-52 mg/l of nitrate and 64-94 mg/l of phosphorus with a pH range of 3.92-4.99.

If this wastewater is not properly treated before it is discharged into the aquatic environment, it can be harmful to the environment and human life [9]. Electrochemical oxidation for wastewater treatment has been studied since the 19th century [10]. The activated oxidation process like photoelectrochemical oxidation forms highly reactive radicals such as hydroxyl radical (HO •). This hydroxyl radical (HO •) has an adequate effect on water purification and removes a variety of persistent toxic compounds. Different studies are showing to focus on reduced toxicity and increased biodegradability [11, 12]. UV/H_2_O_2_ processes in the presence of HO • scavengers and UV radiation absorbers such as dissolved organics (DOM), anions, and reaction intermediates [13]. In electrochemical oxidation, the anode undergoes oxidation, and the cathode is reduced. It focuses on an overview of electrochemical reactors for water and wastewater treatment. The electrochemical system consists of at least two electrodes (anode and cathode and an intermediate region filled with electrolytes). A reference electrode for electrochemical characterization can be added to the system [14]. Electrooxidation was found to be limited in removal in terms of nitrates and phosphates as the maximum pollution mitigation values. The electrochemical oxidation method was environmentally friendly technology which does not generate smock during oxidation-reduction reaction of operation and could not pollute environment during treatment of wastewater contaminants. As a result, it uses an electric current to treat large amount of wastewater with in short period of time [15]. The removal rate was improved by applying UV/H_2_O_2_ to the electrochemical oxidation process. According to [16], they present some of the basic concepts of photoelectrochemical oxidation (PECO) to illustrate the results of higher removal efficiency than electrochemical oxidation, as follows. (1) Hydroxyl radicals can be generated as UV/H_2_O_2_ in the photochemical system. (2) pH, temperature, contact time, and chemical reactivity are all factors that affect the efficiency of H_2_O_2_ treatment. Inorganic substances generally react faster with H_2_O_2_ than organic substances, and the restriction of mass transfer slows down the reaction of organic trace elements. Oxidation by H_2_O_2_ alone is ineffective when using large quantities of certain refractory materials. H_2_O_2_ is also used in surface treatments to clean the surface. H_2_O_2_ is activated by UV light and produces hydroxyl radical a powerful oxidant. Activation of H_2_O_2_ by salt is used in the oxidation process.

The objective of this research is to investigate the effects of Uv/H_2_O_2_ on photoelectrochemical processes with various parameters such as pH, time, current, and electrolytes on the phosphate and nitrate removal from coffee processing wastewater.

## 2. Materials and Methods

### 2.1. Equipment and Chemicals Used

Beaker, magnetic stirrer (model RHB2), desiccator, drying oven, filter paper, (Al-Al), DC power supply (WYJ-o-15V/5A), spectrophotometer (model 6700), vacuum pump, vacuum hood, millimeter, heaters, conical flasks, pH meter, spectrophotometer, standard flasks, Erlenmeyer flasks, measuring cylinder, plastic bottles, burettes, thermometer, funnel, suction flask, wash bottle, porcelain dish, weighing balance (model PW-124), filtration apparatus, graduated cylinder, turbidity meter (Wag-WT3020), pH meter (pH 3310), conductivity meter (Cond 3110), and ultraviolet (UV) lamp (model PUV-1022, Heraeus) were the equipment used for the investigation of samples throughout the experiment. Chemicals used for coffee processing wastewater treatment and analyses such as mercury sulfate (HgSO_4_), ferrous ammonium sulfate (Fe(NH_3_)SO_4_), silver sulfate (Ag_2_SO_4_), ferroin indicator (Fe(o-phen)_3_SO_4_), potassium dichromate (K_2_Cr_2_O7), and sulfuric acid (H_2_SO_4_) are used for COD, hydrogen peroxide (H_2_O_2_) is an oxidizing agent, and the supporting reagents (catalyst) used for the treatment were sodium sulfate (Na_2_SO_4_), KOH, NaOH, HCl, sodium hydrogen carbonate (NaHCO_3_), phenolphthalein, stannous chloride, ammonium molybdate, phenol, buffer solutions, and distilled water.

### 2.2. Sample Collection

About 200 L of wastewater has been taken from Jimma Zone, Yebbu town, coffee processing wastewater discharge point by plastic jerry cans for three days according to wastewater sampling procedure and methods [17]. The canister was soaked in 10% HCl for 24 hours which is used to clean sample holder jerry can, then thoroughly washed and rinsed with distilled water. Plastic boxes were used to protect samples from sunlight and allowed at temperature of 4°C to be maintained during transport. The sample is transported to the laboratory according to the preservation of samples for characterization [18]. Before treating coffee processing wastewater, the waste was filtered to remove floating materials such as coffee seed, coffee pulp, and leaves to allow UV light transmission through the wastewater. As described by [19], the sample was filtered through filter paper and prepared for analysis on the performance of the combined ECO/UV/H_2_O_2_ and electrochemical oxidation process (ECO).

### 2.3. Characterization of Coffee Processing Wastewater

Physicochemical parameters were analyzed in the Water Quality Laboratory, Department of Environmental Engineering, Jimma University. Coffee processing wastewater before treatment was characterized as shown in Table 1, including color, temperature, and chemical parameters associated with the organic content and nutrients such as phosphates and nitrates.  Table 2 describes about experimental and statistical design.

### 2.4. Experimental Design

Figure 1 schematically shows the hybrid electrochemical oxidation process and the experimental analysis setup for UV/H_2_O_2_. The experimental equipment consists of an electrochemical reactor and a UV lamp. UV/H_2_O_2_ processing experimental equipment, a 1 L batch reactor mixed with a magnetic stirrer equipped with a rotating loop and a magnetic rod, was used for the UV/H_2_O_2_ experiment. The loop contains Edan 18 W low-pressure UV. For analysis, 1 liter of wastewater from coffee processing was measured and collected. Next, the pH, time, and current were adjusted, and the electrolyte CaCl_2_ was added, depending on the test design shown in Table 1. Wastewater was analyzed for nitrates and phosphates by inserting the working electrode, reference electrode, counter electrode (Al), and pipette (for blow) into the holes in the rubber stopper.

### 2.5. Experimental Statistical Design

Response surface methodology (RSM) is a method for optimizing affected reactions based on pH, time, current, and electrolytes and is several strategies for finding optimal operating conditions using experimental methods [21, 22]. In this study, laboratory experiments were carried out in the photoelectrochemical oxidation process.

### 2.6. Statistical Data Analysis

Analysis of the data obtained from the laboratory by using empirical formulas was given in [24]

(1) $$\begin{array}{c} \%\text{Nitrate removal}=\frac{{\text{NO}}_{3}\text{i}-{\text{NO}}_{3}\text{t}}{{\text{NO}}_{3}\text{i}}*100 \end{array}$$

where NO_3_i and NO_3_t are the concentrations of nitrate before treatment and after treatment, respectively%.

(2) $$\begin{array}{c} \text{Phosphate removal}=\frac{{\text{PO}}_{3}\text{i}-{\text{PO}}_{3}\text{t}}{{\text{PO}}_{3}\text{i}}*100 \end{array}$$

where PO_3_i and PO_3_t are concentrations of phosphate before treatment and after treatment, respectively.

Phosphate was determined by the stannous chloride method and nitrate by diazotization method (APHA Standard Method-20th Edition).

## 3. Results and Discussions

### 3.1. Effect of pH

The pH value of the solution plays a decisive role in the removal of contaminants in the ECO and UV/H_2_O_2_ processes. As shown in Figure 2, the efficiency of nitrate and phosphate removal was inadequate at low pH 5, but the pH increased to reach neutral pH 7. Depending on the nature of the pollutants, the best pollutant removal is found near pH 7 [22, 25].

According to [26], the pH between 4 and 9 was a major factor in the removal of pollutants. The modified integration of NaOH or H_2_SO_4_ solutions in the pH ranges 5-9 to assess the effect of pH values on process performance [27]. As shown in Figure 3, UV/H_2_O_2_ improves removal efficiency by increasing the destruction of contaminants by the use of powerful substances, so the combination of UV/H_2_O_2_ and ECO is at pH 5-9. The removal efficiency has been further improved. Hydrogen peroxide showed a good ability in reducing bonded chlorides in both organic and inorganic compounds present in the wastewater. Hydrogen peroxide has been used in different experiments to improve the oxygen supply and oxidation rate of suspended and dissolved particles that cause pollution in such water effluent [28]. The effect of pH with COD, color, nitrate, and phosphate % removal potency is shown in Figures 2 and 3.

### 3.2. Effect of Time

The sludge structure affects pollutant removal efficiency. Since, the structure of the sludge may change over time, efficiency of pollutant removal, and floc's settleablity. Figures 4 and 5 show that very long reaction times result in lower removal percentages because very long reaction time leads to metal hydroxide sequestration. In the case of coffee processing wastewater treatment, long time and very short times have low removal efficiency. As a result, 40 minutes is the optimum removal time. As a result, 40 minutes happens to be the optimum removal occasion. According to [29], COD and turbidity treatment efficiency were maximum with an electrolysis time of 30-45 minutes. As shown in Figure 5, the UV/H_2_O_2_/ECO combination improves separation efficiency.

### 3.3. Effect of Current

Figure 6 shows that very depressed current and very high current have reduced removal efficiency concerning all impurities. The best removal efficiency takes place at 0.4 A. In actuality, the current was proportional to potential; as the current grew, so did the amount of usually metallic dissolve; this promotes the formation of Al(OH)_3_ hydroxides. The effectiveness of organic burning decreases when a higher voltage is applied causing oxygen evolution to occur. When the process exists carried out at higher voltages, still, poisoning products made at the anode surface are oxidized. Extremely extreme current negatively affects (decreases) ahead of the treatment of wastewater from the hot beverage made from beans of a tree industry. Electric current is one of the most influential factors in electrochemical processes [30]. Electric current is usually one of the most useful factors in facilitating the electrochemical oxidation process through kinetics. It is important to understand that increasing the current does not necessarily increase the oxidation efficiency. The effect of current on the treatment level depends on the characteristics of the wastewater being treated. On the other hand, the use of higher current generally results in higher operating costs due to the increase in energy use [31].

Figure 6 shows the effect of the current on the removal efficiency with CaCl_2_, and Figure 7 shows that the addition of hydrogen peroxide improves the removal efficiency over the ECO without it.

### 3.4. Effect of Electrolyte

To increase the generated power of the water or wastewater to be concerned, the presence of carbonate or sulfate ions causes the moisture in the air or falling from the sky of Ca^2^+ or Mg^2^+ ions on the electrodes' surfaces, making an insulating layer. Higher electrolyte concentrations reduce energy habits. In the AO and AO-H_2_O_2_ processes, natural compound elimination and mineralization take place more quickly fashionable in the presence of NaCl or CaCl_2_ than fashionable in the absence of Na_2_SO_4_ [32]. The service between electrodes would be to a large extent increased by this insulating coating, resulting in a meaningful reduction in fashionable current efficiency. Because of the increase in generated power, the addition of CaCl_2_ would in addition result in a decline in power custom. Furthermore, chlorine produced electrochemically has been shown to be a useful fashionable water disinfection. As a result, for the tests, an aggregation of 0.5–2.5 g/l CaCl_2_ was used. When distinguished from the other components, the amount of electrolyte determinant has a substantial impact on response.

This happens because CaCl_2_ raises the generated power of the EO system, which makes or becomes better the removal of percent nitrate and phosphate. Due to the extreme ions +2 (CaCl_2_), CaCl_2_ produces a more efficient result than additional cations like NaCl. The addition of a supporting electrolyte (CaCl_2_) happens to boost the solution's generated power [33]. The most widely referenced model of mediated electrochemical oxidation comes from the effect of chlorides on the corrosion of organic matter. Chloride is commonly found in most wastewater streams and is undoubtedly oxidized to chlorine by many types of odorants [34]. By adding the appropriate amount of electrolyte, the output of the generated wastewater was assumed to be the correct value. If the anode potential is extremely enough, a secondary reaction can occur, which is some direct oxidation of the natural molecules present in the leachate with Cl ions. Among the powerful advanced decay techniques, the unintended electrooxidation process is a viable alternative to microscopically destroying large amounts of weight, especially eliminating contaminants, and high conductivity wastewater conditions. It will be a promising technology using powerful oxidants to destroy the natural load of these processes (ACS) [35]. Electron transfer to the anode (reaction (3)) produces ACS from chloride in the water and communicates with water to produce hypochlorous acid (kickback (4)). The equilibrium between hypochlorous acid and the hypochlorite ion in water is powerless in terms of concentration and pH after the speciation of elements in the water. Next to this active class is reaction (5), where chloride radicals are triggered by direct oxidation of the anode reaction (6) [36].

(3) $$\begin{array}{c} 2\text{C}{\text{l}}^{-}⟶{\text{Cl}}_{2\left(\text{aq}\right)+}\left(2{\text{e}}^{-}\right) \end{array}$$

(4) $$\begin{array}{c} {\text{Cl}}_{2}+{\text{H}}_{2}\text{O}⟶\text{HClO}+\text{C}{\text{l}}^{-}+{\text{H}}^{+} \end{array}$$

(5) $$\begin{array}{c} \text{HClO}↔{\text{ClO}}^{-}+{\text{H}}^{+} \end{array}$$

(6) $$\begin{array}{c} {\text{Cl}}^{-}⟶\text{Cl}+{\text{e}}^{-} \end{array}$$

Thus, the generated chlorine gas can oxidize pollutants. It is clear that, for aluminum, the energy consumption is higher and electrode consumption is lower. It is observed that higher conductivity favors high process efficiency.  Figure 8 describes the effect of electrolyte concentration on removal efficiency by using CaCl_2_, and Figure 9 describes the effect of electrolyte on removal efficiency by using UV/H_2_O_2_ and CaCl_2_.

The removal rate of color, COD, nitrate, and phosphate increases with an increasing dose of g/l electrolyte, and the maximum amount of electrolyte is no longer important for removal efficiency. With current amplifiers, this is because the oxidation of organic compounds occurs directly on the electrode surface. The variables are chosen to have maximum nitrate and phosphate removal rates for the best removal performance under weak operating conditions. As shown in Table 3, the targeting principles for the five independent variables include political maintenance time, a mixture of liquid and another substance, pH, current, and salt aggregation in range states. Optimal values for the independent variable are obtained as follows: *pH* = 7, reaction time 40 minutes, energy flow 0.4 amps, and salt concentration 1.5 g/l CaCl_2_. Under these conditions, the level of desirability of the model was effective.

## 4. Conclusions

This study was used to analyze the effects of experimental planning parameters such as initial color, turbidity, COD, phosphate, and nitrate concentrations, and the initial pH, electrolyte mass, contact time, and current of coffee-treated wastewater are possible. Optimized for as high a distance as possible to achieve. The removal of these contaminants depends on pH, time, current, and electrolytes, and H_2_O_2_ has significantly improved removal efficiency. Research results have shown that removal efficiency increases with increasing current, time, electrolytes, and pH, but removal efficiency decreases after optimal levels of these parameters. Second, the combination of electrochemical oxidation and UV/H_2_O_2_ improves the removal efficiency of the photoelectrochemical oxidation process. In this method of treating wastewater from coffee treatment, the independent variable has the greatest impact on improving pollutant removal efficiency. These variables controlled the removal efficiency of the procedure as a function of time length and dose level. The combination of maximum electrochemical oxidation removal efficiency and UV/H_2_O_2_ with CaCl_2_ removes COD, color, turbidity, nitrates, and phosphates at 99.992%, 99.898, 99.898%, 99.22%, and 99.982, respectively. Maximum efficiency is obtained. Optimal results were obtained at pH 7, electrolysis time 40 minutes, current 0.4 amps, and electrolyte 1.5 g CaCl_2_.

## Figures and Tables

**Figure 1:** The experimental setup for photoelectrochemical oxidation [20].

**Figure 2:** The effect of pH on removal efficiency by using CaCl_2_.

**Figure 3:** The effect of pH on removal efficiency by using UV/H_2_O_2_ and CaCl_2_.

**Figure 4:** The effect of time on removal efficiency by using CaCl_2_.

**Figure 5:** Effect of time on removal efficiency by using UV/H_2_O_2_ and CaCl_2_.

**Figure 6:** The effect of current on removal efficiency by using CaCl_2_.

**Figure 7:** The effect of current on removal efficiency by using UV/H_2_O_2_ and CaCl_2_.

**Figure 8:** The effect of electrolyte concentration on removal efficiency using CaCl_2_.

**Figure 9:** The effect of electrolyte on removal efficiency by using UV/H_2_O_2_ and CaCl_2_.

**Table 1:** Raw coffee processing wastewater composition.

S/N	Contaminant	Contents
1	Temperature	43°C
2	Color	Brown
3	Turbidity	144.5 NTU
4	Nitrate	23.5 mg/L
5	Phosphate	9.2 mg/L

**Table 2:** Experimental statistical design [22, 23].

Factor	Name	Units	Type	Minimum	Maximum	Coded low	Coded high	Mean	Std. dev.
A	pH		Numeric	5.00	9.00	-1 ↔ 5.00	+1 ↔ 9.00	7.13	1.57
B	Time	min	Numeric	20.00	50.00	-1 ↔ 30.00	+1 ↔ 50.00	40.00	10.50
C	Current	amp	Numeric	0.2000	0.6000	-1 ↔ 0.30	+1 ↔ 0.50	0.4033	0.0928
D	Electrolyte	g	Numeric	0.5000	2.50	-1 ↔ 1.00	+1 ↔ 2.00	1.50	0.4549

Note: the arrow “↔” represents the range between lower and higher values.

**Table 3:** The characteristics of coffee processing wastewater treated by photoelectrochemical oxidation.

Treatment designs	Major pollutants	CPWW before treatment	CPWW after treated	Removal efficiency (%)	Permissible WHO standard for effluents
ECO/CaCl_2_	Nitrate (mg/L)	23.21	2.243	90.334	5 mg/L
	Phosphate (mg/L)	9.21	0.658	92.855	5 mg/L
ECO/CaCl_2_ and UV/H_2_O_2_	Nitrate (mg/L)	23.21	0.041	99.823	5 mg/L
	Phosphate (mg/L)	9.21	0.008	99.982	5 mg/L

## Data Availability

The data used to support the results of this study are included in the article.
